The article "Rapid response to systemic bevacizumab therapy in recurrent respiratory papillomatosis" was published in 2014. Journal: Oncol Lett.

# Rapid response to systemic bevacizumab therapy in recurrent respiratory papillomatosis

**DOI:** 10.3892/ol.2014.2486

**Published:** 2014-08-28

**Authors:** MICHAEL MOHR, CHRISTOPH SCHLIEMANN, CHRISTOPH BIERMANN, LARS-HENNING SCHMIDT, TORSTEN KESSLER, JOACHIM SCHMIDT, KARSTEN WIEBE, KLAUS-MICHAEL MÜLLER, THOMAS K. HOFFMANN, ANDREAS H. GROLL, CLAUDIUS WERNER, CHRISTINA KESSLER, RAINER WIEWRODT, CLAUDIA RUDACK, WOLFGANG E. BERDEL

**Affiliations:** 1 Department of Medicine A, Hematology, Oncology and Pneumology, University Hospital Muenster, Muenster, Germany; 2 Department of Thoracic Surgery, University Hospital Muenster, Muenster, Germany; 3 Department of Pathology, University Hospital Muenster, Muenster, Germany; 4 Department of Otorhinolaryngology, University Hospital Essen, Essen, Germany; 5 Department of Otorhinolaryngology, University Hospital Ulm, Ulm, Germany; 6 Department of Pediatric Hematology/Oncology, University Hospital Muenster, Muenster, Germany; 7 Department of Pediatrics, University Hospital Muenster, Muenster, Germany; 8 Department of Otolaryngology/Head and Neck Cancer, University Hospital Muenster, Muenster, Germany

**Keywords:** bevacizumab, papillomatosis, anti-angiogenesis

## Abstract

Recurrent respiratory papillomatosis (RRP) is a primary benign disease, which is characterized by papillomatous growth in the respiratory tract. Malignant transformation occurs in only 3–5% of cases, however, local growth of the benign papillomas is interpreted as clinically malignant in a markedly higher proportion of patients. Local surgical or endoscopic interventional debulking or excision is currently the commonly selected treatment method and antiviral therapy is a potential adjuvant approach. However, the long-term management of RRP patients, who commonly require multiple procedures over numerous years, is challenging and the overall therapeutic armamentarium remains unsatisfactory. The administration of systemic bevacizumab treatment in a series of five patients with long histories of RRP, who required repeated local interventions to control papilloma growth is evaluated. Treatment with the anti-vascular endothelial growth factor (VEGF) antibody bevacizumab was administered at a dose of 5 mg/kg (n=1), 10 mg/kg (n=3) or 15 mg/kg (n=1) intravenously to the five RRP patients, who were clinically classified as exhibiting progressive disease. Endoscopic evaluations were performed prior to the first infusion of bevacizumab and intermittently at variable time points during the course of therapy. Histopathological analyses were performed using pre- and post-treatment papilloma biopsies, including immunohistochemical analyses of VEGF and phosphorylated VEGF receptor (VEGFR)-2 expression. The patients received between three and 16 courses of bevacizumab (median, six courses). The first course was initiated when progression following the previous intervention was observed. An immediate response to bevacizumab treatment was demonstrated in all five RRP patients. While the cumulative number of interventions in the five patients was 18 throughout the 12 months prior to the initiation of bevacizumab treatment, only one patient required interventional treatment due to a malignant transformation during the 12 months following treatment with bevacizumab (18 vs. 1 interventions, P=0.042). Histopathological analyses revealed regressive perivascular edema and normalization of the vascular structure, however, immunohistochemical analyses of the VEGF and phosphorylated VEGFR-2 expression did not demonstrate any changes following therapy. Due to the limited number of alternative treatments, VEGF-targeted therapies may represent a promising novel strategy in the treatment of RRP, which may have the potential to modify the current treatment standards, particularly in patients with poorly accessible papilloma lesions, however, this requires further investigation in clinical trials.

## Introduction

Recurrent respiratory papillomatosis (RRP) is a potentially devastating, incurable disease that is caused by infection with the human papilloma virus (HPV), predominantly HPV-6 and -11. Primary benign tumorous manifestations of RRP occur throughout the respiratory tract and may lead to laryngeal, tracheal or bronchial obstructions, and pulmonary nodes and cystic lesions due to valve effects (1). The incidence of RRP in the USA is 4.3/100,000 children and 1.8/100,000 adults (2). Furthermore, malignant transformation occurs in 3–5% of RRP cases (3). When RRP progresses into the pulmonary parenchyma, there are no effective therapeutic strategies and it is almost invariably fatal (3,4). Current standard management of RRP involves repeated local surgical debulking by laser therapy, which is associated with a significant risk of chronic morbidity, including voice mutilation. In total >10,000 interventional treatment procedures for RRP are performed each year in the USA; patients undergo a mean average of 4.4 procedures per year and 19.7 overall (2). The data regarding adjuvant antiviral therapy, particularly intralesional cidofovir, remain inconsistent (5).

A strong mRNA expression of VEGF-A and its receptors, VEGFR-1 and -2 has been observed in tissue samples of RRP patients (6). In 2009, Nagel *et al* (7) reported a case of systemic adjuvant therapy using the anti-VEGF antibody, bevacizumab. In this case, bevacizumab appeared to delay the requirement for further local interventions. In addition, a previous study was conducted, which demonstrated a series of adults exhibiting papillomatosis who were treated with combined laser therapy and sublesionally injected bevacizumab (8); a second study was recently conducted in a population of children (9).

The clinical courses of five patients with long histories of RRP in whom the systemic administrations of bevacizumab were evaluated are reported.

## Patients and methods

### Patient characteristics

Between April 2011 and May 2012 five patients aged 8–56 years (median, 43 years) presented at the Department of Medicine (University Hospital, Muenster, Germany) with histories of RRP ranging between 6 months and 37 years (median, 3 years). The patient characteristics are presented in Table I. The manifestations of RRP were as follows: Lung parenchyma, n=2; tracheobronchial involvement, n=2; the larynx and vocal cords, n=3; and sinonasal inverted papilloma, n=1. All of the patients had previously received multiple local interventions (from three to >30) predominantly by laser therapy. One patient suffering from papilloma involvement of the paranasal sinuses had received a radical surgery by midfacial degloving and adjuvant radiotherapy. One patient, who was exhibiting lung parenchymal involvement, had received a middle lobe resection and demonstrated evidence of malignant transformation of a papilloma manifestation. In addition, the administration of additional adjuvant medical therapeutic agents, such as cidofovir, celecoxib and interferon had been tried in two patients. However, all five patients presented with progressive disease at the time of treatment initiation with systemic bevacizumab therapy. The report is in accordance with the Declaration of Helsinki guidelines.

### Treatment and response evaluation

Written informed consent was obtained from each patient. Bevacizumab administration was initiated at a dose of between 5 and 15 mg/kg intravenously every 2–3 weeks. Treatment intervals were subsequently extended after achieving the maximum response as demonstrated by endoscopy and/or bronchoscopy. Endoscopy was performed prior to and between days three and seven following treatment initiation. Follow-up endoscopies were performed prior to every subsequent course of bevacizumab. Digital endoscopic imaging documentation was conducted using a routine documentation systems (BF Q180 video-bronchoscope; CV-160 video-processor; Olympus Corporation, Tokyo, Japan). Computed tomography (CT) was performed in two patients to follow up the RRP involvement of the lung parenchyma or paranasal sinuses.

### Histopathological analyses

Papilloma tissue samples were obtained for standard histological and immunohistological analyses prior to and following the first infusion of bevacizumab in two patients. For immunohistochemistry, formalin-fixed and paraffin-embedded tissues were analyzed using primary polyclonal rabbit anti-human antibodies specific to VEGF (Santa Cruz Biotechnology, CA, USA; working dilution, 1:50), phosphorylated VEGFR-2 (Santa Cruz Biotechnology; working dilution, 1:50) and the alkaline phosphatase anti-alkaline phosphatase double-bridge technique (DakoCytomation, Glostrup, Denmark). Briefly, tissue sections were deparaffinized in xylene and rehydrated in a graded ethanol series. Following antigen retrieval in a microwave oven at 450 W (twice for 7 min in 10 mM sodium citrate [pH 6.0; DakoCytomation]) the primary antibodies were applied to the tissue sections overnight at 4°C. Subsequent steps were performed according to the manufacturer’s instructions. The Fast-Red substrate (DakoCytomation) was used for detection of phosphatase activity and sections were counterstained with hematoxylin and eosin (Merck KGaA, Darmstadt, Germany).

### DNA fragmentation assay

To investigate apoptosis in the histology specimen, the In Situ Cell Death Detection kit, AP (Roche, Basel, Switzerland) was used, which is based on the Terminal deoxynucleotidyl transferase dUTP nick end labeling (TUNEL)-reaction. TUNEL-positive apoptotic cells were counted in three representative independent microscopic fields (magnification, 200×) per tumor (Axioskope, Zeiss, Oberkochen, Germany).

### Statistical analysis

For statistical analysis the Wilcoxon signed-rank test was used. P-values were two-sided and P<0.05 was considered to indicate a statistically significant difference.

## Results

### Patient 1

This patient was a 43-year-old male, who had been diagnosed with HPV-11-associated respiratory papillomatosis at the age of 6 years. Between the ages of 8 and 13 years, multiple interventions, including a temporary tracheostomy, had been necessary and were followed by a stable disease phase for ~20 years. Since 1997, the disease had begun to progress and required repeated interventions. In April 2011, multiple tracheal papilloma manifestations led to a tracheal stenosis of upto 70%. CT scans revealed numerous pulmonary nodes, cystic lesions and a tumor measuring 2.5×2.6 cm in the middle lobe. Tracheal laser therapy temporarily resulted in good short-term results and resection of the middle lobe with lymphadenectomy led to the diagnosis of a papilloma with transformation to squamous cell carcinoma (T_1b_N_0_M_0_, TNM Classification for Malignant Tumors) (10).

Four weeks later, a follow-up bronchoscopy demonstrated progression of the tracheal papillomatosis and clinical stridor was detected (Fig. 1). At that time, systemic treatment with bevacizumab was initiated at a dose of 10 mg/kg. Three days after treatment initiation a bronchoscopy indicated a significant response, with a reduction of ~50% of the tracheal manifestations and the stridor had disappeared completely. After 21 days, certain papillomas were no longer present, and the dyspnea and hoarseness had improved markedly, prompting the continuation of the bevacizumab therapy. Due to the activity and good tolerability of bevacizumab, it was decided that the patient could be treated at 14-day intervals. Following eight cycles of treatment (day 139) a bronchoscopy demonstrated only minimal residual disease (Fig. 1). The very good partial remission (VGPR), which was also observed in the chest CT-scans (Fig. 2), showed ongoing stability for 27 months at the time of writing. The patient is well and has resumed normal daily activities. The only treatment-associated side-effect was mild hypertension, which was managed with a calcium antagonist. Treatment intervals were extended to 4 months, and no surgical interventions were necessary subsequent to treatment initiation with bevacizumab.

### Patient 2

This 49-year-old male was diagnosed with severe laryngeal RRP in January 2011. At the initial diagnosis local papilloma debulking was achieved using laser therapy. However, 6 months later, the papillomatosis relapsed and required a second laser-based intervention. The disease progressed again and bevacizumab treatment was initiated (dose, 10 mg/kg). An endoscopy prior to treatment revealed exophytic papilloma growth in the right supraglottic area (Fig. 3A). Pathological examination of biopsies taken from the area excluded the presence of squamous cell carcinoma. An endoscopy on day four after the first administration of bevacizumab demonstrated a rapid response in the patient. A second control endoscopy, which was performed immediately prior to the application of the second cycle of bevacizumab on day 20, showed further regression of the papilloma mass (Fig. 3A). In parallel, hoarseness improved significantly within a few days and the patient did not experience treatment-associated side-effects. However, in this case, clinical worsening led to a re-evaluation, including a CT scan prior to the third cycle of bevacizumab, revealing destructive tumor growth that was potentially malignant transformation in the subglottic area, while the supraglottic RRP manifestation demonstrated a sustained VGPR. A laryngectomy was performed and histology identified the co-existence of squamous cell carcinoma and papilloma lesions. At present, the patient has not yet demonstrated a relapse of RRP.

### Patient 3

This patient was a 56-year-old female, who was diagnosed with laryngeal and glottal RRP in 2009. Clinical symptoms predominantly included hoarseness, an irritative cough and dyspnea. Throughout the subsequent 3 years a total of 16 laser ablation therapies were necessary at increasingly shorter intervals, with the final interventions only leading to a short-term improvement of the symptoms. Systemic therapy with bevacizumab was initiated in March 2012. An endoscopy seven days after the first dose of bevacizumab (10 mg/kg) revealed a partial response (PR) of the supraglottic papilloma, while the manifestation on the right vocal cord remained stable. After the second cycle, a further reduction of the supraglottic lesion was observed. Clinically, the patient’s voice became increasingly powerful and dyspnea on exertion significantly improved shortly after treatment initiation. Bevacizumab therapy was paused following four cycles and the patient’s clinical condition remained stable for >9 months (Fig. 3B). After this period the patient developed symptoms of recurrence with an endoscopy indicating recurrence of papilloma growth. Bevacizumab therapy was resumed and resulted in clinical improvement within five days. Again, an endoscopy on day 14 demonstrated the complete resolution of the supraglottic papilloma. One infraglottic lesion, which had not responded to the same extent was treated with additional laser therapy and a diagnosis of malignant transformation was excluded.

### Patient 4

A 2-year-old female, who was diagnosed in 2007 with HPV-11-associated RRP involving the larynx, trachea, deeper bronchi, and the lung parenchyma required a tracheostomy in August 2008 and multiple laser ablation therapies until January 2012. Adjuvant treatment attempts with interferon-alpha, cidofovir and celecoxib did not result in disease control. In January 2012 laser therapy of the large tracheal RRP manifestations was performed. Fig. 3C shows the papilloma lesions in the right main bronchus, which were not locally treated at that time. Two life-threatening airway complications occurred during an elective change of the tracheal cannula and in the context of a tracheal laser intervention. To avoid re-growth of the papillomas in the trachea and disease progression in the right main bronchus the decision to initiate bevacizumab treatment (5 mg/kg every 2 weeks) was made following the laser treatment. After four cycles of bevacizumab no further papilloma growth was observed in the trachea and bronchi, and the treatment was paused (Fig. 3C). Monthly bronchoscopic assessments did not indicate recurrent disease activity for 6 months. Five months after bevacizumab discontinuation, an endoscopy showed multilocular papilloma relapse in the trachea and bronchi, and a fifth cycle of bevacizumab was administered. On day two after administration, a notable response was observed and no further local interventions for papillomatosis were necessary for more than one year of treatment at three-monthly intervals. One solitary manifestation at the distal end of the tracheal cannula was clinically classified as a granuloma and had to be laser abraded (histologically confirmed as papilloma) in May 2013.

### Patient 5

A 32-year-old male was diagnosed with nasopharyngeal papillomatosis and paranasal sinus papilloma in 2010. Over 24 months several interventions, including laser vaporization and radical surgery via midfacial degloving had been necessary. In February 2012 an attempt to treat the sinonasal inverted papilloma with radiotherapy was made. However, three months later additional laser therapy was required and was complicated by chronic bleeding from the nasopharynx, which led to severe anemia (hemoglobin, 5.5 g/dl). A CT scan performed in July 2012 showed inverted papilloma in all of the paranasal sinuses, including a complete obstructed right frontal sinus, a subtotal obstruction of the left frontal sinus and a complete obstruction of the left maxillary sinus. An endoscopy revealed recurrent papilloma growth at the velum (Fig. 3D) while the possibility of deeper tracheobronchial manifestations could be excluded. It was decided that this patient could be treated with bevacizumab at a dose of 15 mg/kg every three weeks. An endoscopy on day four following treatment initiation indicated an immediate response of the papilloma manifestations that were located at the velum; furthermore, a partial remission with a 50% reduction was observed on day 20 (Fig. 3D). A CT scan after three cycles of bevacizumab also revealed a response in the left frontal sinus and the left maxillary sinus, while the right frontal sinus continued to be obstructed (Fig. 2B). The patient experienced no treatment-associated complications. After the third cycle no further regression of the papilloma manifestations at the velum occurred and the treatment was paused. Two months later, a routine endoscopy showed papilloma progression again and a fourth cycle of bevacizumab was administered, which resulted in immediate papilloma regression.

### Histopathological analyses

Histopathological analyses of pre- and post-therapeutic papilloma biopsies showed regressive edema and normalization of the vascular structures (Fig. 4). However, immunohistochemical analyses of the VEGF and phosphorylated VEGFR-2 expression did not show any changes following therapy with bevacizumab (data not shown).

### Summary of clinical efficacy

The clinical efficacy of systemic bevacizumab treatment is summarized in Table II. Bevacizumab induced PR or VGPR of papilloma manifestations in 5/5 patients. When comparing the cumulative number of local interventions during the 12-month period prior to bevacizumab treatment initiation with the 12 month period following bevacizumab treatment, the number of interventions was reduced from 18 to one (P=0.042, Wilcoxon signed-rank test).

## Discussion

The induction of papilloma regression is presented in five consecutive patients with progressive RRP who, following various previous treatment attempts, were administered with systemic bevacizumab therapy at our institution. Previously, systemic administration of bevacizumab has been hypothesized as an effective adjuvant treatment modality following local intervention. It was reported that bevacizumab may have delayed relapse in one case of RRP (7) and was reported to potentially improve photoangiolytic laser therapy, when used concomitantly and applied topically (8,9). In addition, epidermal growth factor receptor inhibition using gefitinib or erlotinib demonstrated efficacy in two cases of RRP (11,12).

An immediate and sustained therapeutic effect of systemically administered bevacizumab was observed in all five RRP patients in the present case series. Notably, it was possible to document the response to treatment bronchoscopically as early as within a few days following the first infusion of bevacizumab. Continued anti-VEGF treatment resulted in sustained PR or VGPRs of tracheal or laryngeal papilloma manifestations. Remission has been sustained in one patient via administration of bevacizumab at prolonged treatment intervals of 3–4 months. Three patients, who exhibited disease progression following discontinuation of bevacizumab, subsequently responded again following the second cycle of treatment. Notably, none of the patients showed papilloma progression whilst treatment was ongoing. Patient 2 required a laryngectomy due to malignant transformation. The condition of patient 3 was clinically stable for 9 months following bevacizumab treatment, however, papilloma regrowth was observed following treatment discontinuation. After this re-growth, re-treatment led to a complete resolution of the supraglottic lesions. In this patient, an infraglottic lesion did not respond to the same extent as the other lesions and was abrased; a diagnosis of malignant transformation was excluded. In patient 4, with former multilocular tracheobronchial and lung parenchyma involvement, a solitary manifestation, which was clinically interpreted as granuloma associated with mechanical irritation by the distal end of the tracheal cannula, had to be abrased. However, histological assessment indicated that this particular manifestation was papilloma growth.

At the time of writing the longest period of progression-free survival observed during follow-up is 27 months in patient 1, who is receiving maintenance therapy. Notably, in the present case series, it was possible to document the responses to bevacizumab therapy with regard to lung parenchyma involvement and papillomas of the paranasal sinuses, which are usually not accessible to local interventions (Fig. 2).

The rapid response to bevacizumab was accompanied by a disappearance of the perivascular edema in papilloma lesions as revealed by histopathological analyses of the pre- and post-treatment papilloma lesions. This finding is consistent with the antibody-mediated inhibition of VEGF-induced vascular permeability (13). DNA fragmentation assays that were performed on papilloma tissues to detect apoptosis did not indicate significant differences prior to and following the administration of bevacizumab. This indicates that the observed therapeutic effect is predominantly mediated by modulation of the vasculature and not by induction of apoptosis.

In conclusion, the experience of the five present patients suggests that systemic bevacizumab presents a highly effective treatment option for RRP, offering a unique opportunity even for patients with non-accessible bronchial lesions, lung parenchyma involvement, papillomas of the paranasal sinuses, or for patients at high risk for voice mutilation by interventional therapies. These findings indicate that systemic bevacizumab treatment may have the potential to alter the current management of RRP. Whether the treatment will have an impact on the frequency of malignant transformation in papillomatosis remains unclear and VEGF-targeted therapeutic strategies require further investigation in clinical trials.

## Figures and Tables

**Figure 1:** Representative bronchoscopic images of the laryngeal (first row) and tracheal (second row) papilloma manifestations in Patient 1. Images in the first column demonstrate the pre-therapeutic condition. On day three, following the first dose of bevacizumab, a significant regression of papilloma lesions was observed (second column) and a very good partial remission with only minimal papilloma residues was documented under continuous bevacizumab treatment on day 139 (third column).

**Figure 2:** (A) Patient 1: Computed tomography (CT) scannings of a pulmonary mass in the left lower lobe prior to and one year after initiation of bevacizumab treatment. (B) Patient 5: CT of the (a) left maxillary sinus and (b) left frontal sinus that were initially obstructed by inverted papilloma and were cleared following three cycles of bevacizumab therapy.

**Figure 3:** Bronchoscopic images of papilloma manifestations. (A) Patient 2: Laryngeal papilloma manifestations prior to bevacizumab (left), on day four following administration of bevacizumab (middle) and on day 20 under continuation of systemic bevacizumab treatment (right). (B) Patient 3: Supraglottic papilloma lesion prior to administration of bevacizumab (left) and on day 158 (right). (C) Patient 4: Papilloma manifestations in the right main bronchus prior to (left) and on day 180 following initiation of bevacizumab therapy (right). (D) Patient 5: Papilloma located on the velum prior to (left), on day four (middle) and on day 20 following the first administration of bevacizumab (right).

**Figure 4:** Histopathological changes following bevacizumab therapy. Biopsies obtained (A) prior to and (B) following bevacizumab therapy (four cycles) reveal a marked decrease of perivascular edema (stain, hematoxilin and eosin; magnification, ×200).

**Table I:** Patient characteristics.

Patient	Age at initial diagnosis (years)	Gender (M/F)	Total debulking interventions pre-bevacizumab	Age at treatment initiation (years)	Cycles (n)
1	6	M	>30	43	16
2	49	M	2	49	3
3	53	F	16	56	6
4	2	F	>30	8	9
5	32	M	6	34	6

M, male; F, female.

**Table II:** Summary of the clinical efficacy of systemic bevacizumab treatment.

Case	Best response	Freedom from progression following treatment discontinuation (months)	Second response following treatment discontinuation and progression	No. of interventions in 12 months	

				Prior to bevacizumab	Following bevacizumab
1	VGPR	>4	N.a.	3	0
2	PR	N.a.	N.a.	2	1^a^
3	VGPR	9	Yes	6	0
4	VGPR	5	Yes	3	0
5	PR	2	Yes	4	0
All	-	-	-	18	1^b^

a Laryngectomy for malignant transformation.

b P=0.042.

VGPR, very good partial remission; PR, partial response; N.a., not applicable.

## References

[1] Glikman D, Baroody FM (2005). Images in clinical medicine. Recurrent respiratory papillomatosis with lung involvement. New Engl J Med.

[2] Derkay CS, Wiatrak B (2008). Recurrent respiratory papillomatosis: a review. Laryngoscope.

[3] Kimberlain DW (2004). Current status of antiviral therapy for juvenile-onset recurrent respiratory papillomatosis. Antiviral Res.

[4] Gélinas JF, Manoukian J, Côté A (2008). Lung involvement in juvenile onset recurrent respiratory papillomatosis: a systematic review of the literature. Int J Pediatr Otorhinolaryngol.

[5] Chadha NK, James A (2010). Adjuvant antiviral therapy for recurrent respiratory papillomatosis. Cochrane Database Syst Rev.

[6] Rahbar R, Vargas SO, Folkman J (2005). Role of vascular endothelial growth factor-A in recurrent respiratory papillomatosis. Ann Otol Rhinol Laryngol.

[7] Nagel S, Busch C, Blankenburg T, Schütte W (2009). Treatment of respiratory papillomatosis - a case report on systemic treatment with bevacizumab. Pneumologie.

[8] Zeitels SM, Barbu AM, Landau-Zemer T (2011). Local injection of bevacizumab (Avastin) and angiolytic KTP laser treatment of recurrent respiratory papillomatosis of the vocal folds: a prospective study. Ann Otol Rhinol Laryngol.

[9] Rogers DJ, Ojha S, Maurer R, Hartnick CJ (2013). Use of adjuvant intralesional bevacizumab for aggressive respiratory papillomatosis in children. JAMA Otolaryngol Head Neck Surg.

[10] Sobin LH, Gospodarowicz MK, Wittekind C (2009). TNM Classification of Malignant Tumours.

[11] Limsukon A, Susanto I, Hoo GW (2009). Regression of recurrent respiratory papillomatosis with celecoxib and erlotinib combination therapy. Chest.

[12] Bostrom B, Sidman J, Marker S (2005). Gefitinib therapy for life-threatening laryngeal papillomatosis. Arch Otolaryngol Head Neck Surg.

[13] Ferrara N (2005). VEGF as a therapeutic target in cancer. Oncology.

